RETRACTED

# Biometric Recognition of Finger Knuckle Print Based on the Fusion of Global Features and Local Features

**DOI:** 10.1155/2022/6041828

**Published:** 2022-01-07

**Authors:** Wenwen Li

**Affiliations:** College of Mechanical Engineering, Baicheng Normal University, Baicheng 137000, China

## Abstract

Compared with the most traditional fingerprint identification, knuckle print and hand shape are more stable, not easy to abrase, forge, and pilfer; in aspect of image acquisition, the requirement of acquisition equipment and environment are not high; and the noncontact acquisition method also greatly improves the users' satisfaction; therefore, finger knuckle print and hand shape of single-mode identification system have attracted extensive attention both at home and abroad. A large number of studies show that multibiometric fusion can greatly improve the recognition rate, antiattack, and robustness of the biometric recognition system. A method combining global features and local features was designed for the recognition of finger knuckle print images. On the one hand, principal component analysis (PCA) was used as the global feature for rapid recognition. On the other hand, the local binary pattern (LBP) operator was taken as the local feature in order to extract the texture features that can reflect details. A two-layer serial fusion strategy is proposed in the combination of global and local features. Firstly, the sample library scope was narrowed according to the global matching result. Secondly, the matching result was further determined by fine matching. By combining the fast speed of global coarse matching and the high accuracy of local refined matching, the designed method can improve the recognition rate and the recognition speed.

## 1. Introduction

Hand-based multibiometric recognition system occupies an important position in the field of biometric recognition. Compared with the most traditional fingerprint identification, knuckle print and hand shape are more stable, not easy to abrase, forge, and pilfer; in aspect of image acquisition, the requirement of acquisition equipment and environment are not high; and the noncontact acquisition method also greatly improves the users' satisfaction; therefore, finger knuckle print and hand shape of single-mode identification system have attracted extensive attention both at home and abroad. A large number of studies show that multibiometric fusion can greatly improve the recognition rate, antiattack, and robustness of the biometric recognition system. However, multifeature fusion undoubtedly increases the computational complexity, feature dimension, and computation time. Therefore, the bimodal feature recognition system proposed in this paper presents a new solution to this problem. The hand shape feature is stable in a period of time, which has strong anticounterfeiting and anti-attack performance; the feature extraction algorithm is simple, and the recognition speed is high; and the finger knuckle print is rich in textures, just like fingerprints, which can remain stable for a long time and contain high individual differences. The fusion of the two features can achieve complementary advantages and improve the recognition accuracy, stability, and antiattack performance of the biometric identification system.

RETRACTED

Finger knuckle print, as a biological feature, constitutes a unique texture feature of human hands together with fingerprint and palm print. There is no commercial biometric recognition system based on finger knuckle print, and the research results of finger knuckle print recognition are quite a few. Most of the existing finger knuckle print research results are based on the outer knuckle images of opisthenar. Lin Zhang et al. from Hong Kong Polytechnic University had designed the dorsal digital joint collection device, which was small in size, simple, and portable. Besides, they had used this device to establish the finger knuckle prints database, including 660 finger images from 165 volunteers; 12 images were collected from each of the 4 fingers other than the thumb from each person; and a total of 7,920 images were included in the database) [1]. At the finger knuckle print recognition stage, Zhang et al. had proposed a new method to extract the area of interest (ROI) of finger knuckle print, which could extract ROI through localizing the *X*-axis and *Y*-axis of the image; besides, at the feature extraction phase, the direction information was extracted using the Gabor filter-based improved competitive code, and the amplitude code was proposed to extract the amplitude information, followed by fusion of these two features for matching at last [2]. Zhang et al. had utilized the Gabor filter to extract the image direction information as the local feature; at the same time, the Fourier transform coefficient was extracted as the global feature. At the feature matching phase, the matching distances of local and global features were calculated; eventually, the two distance fusion results were used as the final identification results [3]. Shoichiro Aoyama et al. had collected the finger knuckle print image on the lateral phalangeal joint surface and proposed the local block matched band-limited phase-only correlation (BLPOC) algorithm [4].

However, the inner finger knuckle print can be recognized by the same acquisition equipment as the hand shape and the palm print from the perspective of image acquisition. In other words, the inner finger knuckle print is more easily integrated with the features of the hand shape and the palm print and constitutes a multifeature biometric recognition system to improve the accuracy of biometric recognition [5]. Therefore, this paper collected the inner finger knuckle print image for biometric recognition. The inner finger knuckle print is shown in Figure 1(a), and the corresponding ROI is shown in Figure 1(b).

RETRACTED

In general, features extracted in the feature extraction process can be divided into global features and local features. (1) Global feature-based method: principal component analysis (PCA), linear discriminant analysis (LDA), independent component analysis (ICA), discrete cosine transform (DCT), and discrete Fourier transform (DFT) were used to recognize face and finger knuckle print. In particular, PCA and LDA have become the most commonly used global feature extraction methods in the field of biometric feature recognition [6, 7]. (2) Local feature-based method: LBP and Gabor wavelet are used [8, 9]. Global and local features have been extensively utilized, and the fusion of the two has also been used in face recognition and dorsal digital joint print recognition [9, 10]. For instance, Zhang et al. had adopted the Gabor filter to extract the image direction information as the local feature, while the Fourier transform coefficient as the global feature; at the matching phase, the matching distances of local and global features were calculated, respectively, and the fusion result of these two distances was used as the final identification result. An improved feature extraction method called average line local binary pattern (ALLBP) is introduced by Bahmed Farah to improve feature extraction of this region of the inner print of the finger [11]. Vidhyapriya has proposed a method for secure biometrics authentication using finger knuckle print (FKP). The texture patterns from finger knuckle are extracted using Gabor with exception-maximization (EM) algorithm, and the feature vectors from these texture patterns are acquired using scale invariant feature transform (SIFT) algorithm [12]. These algorithms have achieved satisfactory results. However, few literatures focus on the fusion of both global and local features. For image identification, global and local features have represented the different properties of the image, both of which are of great importance. Specifically, the global feature describes the overall feature, which is more suitable for crude extraction, while the local feature depicts the image details, which is essential for texture and suitable for detail distinguishing. The importance of these two features cannot be evaluated separately; therefore, the global feature should be used in combination with the local feature to comprehensively utilize the advantages of the two in terms of image identification. This was the major starting point of the finger knuckle print recognition in this paper. Therefore, the global combined with local feature extraction method was adopted in the finger knuckle print recognition in this paper.

RETRACTED

## 2. Database Construction

A hand image acquisition device is designed, which can acquire hand shape and finger knuckle print images at the same time in one acquisition, and a full-hand image database is established.

One hundred volunteers of different genders and different ages were selected, and each of them was collected 5 times at different time periods on different dates. Three images were collected each time, and 15 images were obtained for each person, and a database of 1,500 images was obtained. According to the proposed image preprocessing method, a finger knuckle print ROI database is established to verify the effectiveness of the proposed algorithm. According to the extraction method of finger knuckle print region of interest (ROI) presented in [13], a finger knuckle print database is constructed, and there are 1,500 sets of finger knuckle print in the database. Some examples of the image are shown in Figure 2. Four sets of images represent index finger, little finger, middle finger, and ring finger [14]. Every line of images represents finger knuckle prints of one finger acquired at different times, and two lines represent finger knuckle prints of different volunteers.

## 3. Feature Extraction

### 3.1. Global Feature Extraction

The global features of finger knuckle print were extracted through PCA. There are 65,536 (256 ∗ 256) pixel values in a normalized finger knuckle print ROI image. Each pixel value represents a feature of the image. An image can be represented by a 65,536-dimension column vector. According to the idea of PCA, a new coordinate system can be established, and a low-dimensional feature vector represents the original image. This dimensionality reduction method can not only decrease the computational complexity but also eliminate the noise interference in uncorrelated features. In a new coordinate space, the eigenvalue size represents the amount of sample information contained in its corresponding feature vector. In descending order, the eigenvector corresponding to the first eigenvalue contains the most information of the sample. Therefore, the feature vectors corresponding to the first few feature values contain most of the sample information [6, 15].

RETRACTED

In the recognition of finger knuckle print, every ROI is a sample in a higher-dimensional space, and the higher dimensional space can be presented as follows:

(1) $$\begin{array}{c} X^{\left(\mu \right)}=\left(\begin{array}{c} X_{1}^{\left(\mu \right)}\\ X_{2}^{\left(\mu \right)}\\ \vdots \\ X_{N}^{\left(\mu \right)} \end{array}\right),\;\mu =1,2,\ldots ,P, \end{array}$$

where *N* is the eigendimension of sample space, that is the number of pixels in the ROI, *P* is the number of samples that is gathered to recognize, and *X*_*N*_^*μ*^ is the *N*-th feature in the *μ*-th images.

As shown in Figure 3, the cumulative contribution rate of the first 200 feature vectors reaches as much as 99%. The sample features represented by the feature vectors are not related to each other since the feature vectors are orthogonal to each other. A new image can be generated from the feature vectors, that is, a feature image. Each feature image represents a unique feature of the sample, and the first feature image contains most of the features. The knuckle image (gray normalized for display) reconstructed from feature vectors of different dimensions is shown in Figure 4. The schematic diagram (gray normalized for display) of the feature image generation is shown in Figure 5. It can be seen that the more features are selected, the closer the reconstructed result is to the original image.

In the existing literature about finger knuckle print recognition, the influence of the four-finger feature weight on the recognition rate is not mentioned in the feature fusion link of four-finger images [1, 6, 8, 10]. Considering that a four-finger image contains different texture details, the weights in the hand recognition should also be different.

Figure 6 shows the relationship between the recognition rate and the feature dimension in the case of different weight ratios for four fingers. The weight ratio is index finger:little finger:middle finger:ring finger. The recognition rate is in direct proportion to the feature dimension. However, when the feature dimension reaches a certain value, its increase will cause information redundancy, thereby decreasing the recognition rate. When the four-finger weights were the same and reached 32 dimensions, the four-finger knuckle print recognition rate could achieve the highest level of 94.4%, as presented in Figure 6(a). When the four-finger weights were not the same, the PCA dimension was greatly reduced to 24 dimensions to reach the same recognition rate of 94.4%, as displayed in Figure 6(b). Moreover, it could be known from Figure 2 that when the PCA feature dimension was changed, the maximal recognition rate was 94.4%. As for the different weights of the four fingers, the PCA dimension will decrease substantially when the recognition rate is the same. The experimental results show that the contributions to the recognition result are different due to the different finger knuckle print of the four fingers. Therefore, the weight ratio cannot be set simply in four-finger image fusion recognition.

RETRACTED

Due to the different weights of the four fingers, the feature dimension is between 20 and 35, and the maximum recognition rate is up to 94.4%. In order to further determine the weight ratios of the four fingers, minimize the feature dimension, and improve the recognition speed, different four-finger weight combinations were selected to obtain the relationship between the weight combination and the corresponding feature dimension when the highest recognition rate was 94.4%, as shown in Table 1.

Table 1 has selected the different four-finger weight combinations so as to obtain the relationship between weight combination and corresponding feature dimension when the highest recognition rate of 94.4% was achieved. As could be found, when the four-finger weight ratio was 2:2:3:2, the highest recognition rate of 94.4% could be obtained in the presence of 21-dimension features. According to the experimental results, the phalangeal configurations of the middle finger contain the most abundant texture information, and the experimental results are also in line with the sensory effects of human eyes.

### 3.2. Local Feature Extraction

In this paper, LBP (local binary mode) was used to extract the texture features of finger knuckle print. IBP is a texture description operator that describes the local features of an image [16]. By comparing the gray value of any point in the image with that of each point in the neighborhood, a binary sequence is generated and multiplied by the corresponding weights to obtain the pixel value of the middle point in the neighborhood as the LBP code. According to the definition of LBP, local texture information can be represented by the gray-scale difference between the neighborhood pixel and the center point. Therefore, the LBP operator has strong robustness to illumination when calculating the texture information, and the LBP histograms under different illumination conditions are consistent. An LBP operator has a variety of deformations according to different needs, such as a circular rotation invariant LBP operator and an LBP operator with unified mode. This paper selects a circular window with *P*=8 and *R* = 2, as shown in Figure 7 [16–19]. The LBP operator with a unified mode is calculated, and each sub-block contains 59 features.

The steps for feature extraction are as follows:

  Step 1. Each ROI image is normalized to a size of 256 ∗ 256.
  Step 2. The image is divided into blocks, and the whole image is divided into 16 blocks by a 64 ∗ 64 window. The LBP histograms of the local windows are calculated and connected to obtain an eigenvector including 944 values.
  Step 3. The LBP histogram of the near finger knuckle print is connected to form the final histogram feature as the extracted finger knuckle print feature, and its vector dimension is 3,776.

RETRACTED

The ROI images of four-finger knuckle prints under different light conditions are shown in Figure 8. The histogram of two sets of ROI images is shown in Figure 9(a), and the blue histogram represents the images that are brighter, while the red histogram represents the images that are darker.  Figure 9(b) shows the LBP histogram characteristics of two different collected samples for comparison. It can be clearly seen from the details that there are minor differences among the LBP histograms of the same sample under different illumination, while those of different samples are much greater. It further confirms that the illumination robustness of the LBP operator can be used as a feature extraction method for noncontact biological features, especially texture feature recognition.

To verify the effect of different numbers of selected points and radius on the recognition accuracy rate and recognition time in the LBP operator, this paper had selected the various point numbers *P* and radii *R* of the round LBP operator for comparative experiments, and (*P*, *R*) were selected as (8, 1), (8, 2), (8, 3), (16, 1), (16, 2), and (16, 3). In addition, the ROI images of the four-finger near finger knuckle prints were collected for LBP feature extraction and recognition. The experimental results are displayed in Table 2.

According to the comparison experiment results, when the number and radius of the LBP operators were 8 and 2, respectively, the recognition rate was up to 92.4%. The training time of 800 ROI images was 24.8 s, and the test time of 700 ROI images was 40.68 s. When there were 16 points, the recognition rate decreased, and the training time and test time also multiplied. Obviously, the (8, 2) LBP operator had the best performance in recognition rate and running time.

## 4. Fusion Strategy

Global feature recognition extracts features with low dimensions, which are rough matching. The recognition speed is high but the recognition accuracy is low. However, local feature recognition extracts features with high dimensions, which belongs to fine matching. The recognition rate is great, but the recognition speed is relatively low [20–24]. Therefore, in order to comprehensively utilize the advantages of the two features and improve the recognition rate and recognition speed of the recognition system, this paper adopted the serial fusion strategy to design a two-layer classifier. The first-layer classifier mainly completed the global feature matching in the sample database to be tested. According to the matching result, the test sample library was initially screened, and all images in the database were sorted according to the similarity. The number of samples to be matched was decreased, and the samples with large differences were excluded. The second-layer classifier further identified the remaining samples according to the extracted local features and determined the recognition results. The strategy can reduce the number of fine matching and improve the recognition speed substantially. The matching strategy of global and local fusion is shown in Figure 10.

RETRACTED

The first-layer classifier was a minimum distance classifier. In order to further improve the recognition speed, two fixed thresholds *R*_1_ and *R*_2_ were set in this paper. The Euclidean distance between the two images is *R*. When the Euclidean distance *R* between the image to be detected and the image in the database is smaller than *R*_1_, they belong to the same finger knuckle print. When *R* is greater than *R*_2_, they belong to different finger knuckle print. Therefore, the image of *R* < *R*_1_ or *R* > *R*_2_ will not be screened in the second-layer classifier.

After being screened by the first-layer classifier, the *N* image of *R*_1_ < *R* < *R*_2_ is taken as input to the second-layer classifier. The selection of *R*_1_ and *R*_2_ can also influence the results. The larger the *R*_2_ value, the lower the recognition speed of the second-layer classifier. The smaller the *R*_2_ value, the more likely the image of the same type is excluded. *R*_1_ is selected in the same way. Therefore, it is necessary to find a balance point between the recognition rate and the recognition speed and select an appropriate distance threshold.

The k-nearest neighbor algorithm was used in the second-layer classifier to calculate the chi-square distance between the LBP feature values. The recognition results were obtained according to the distance.

## 5. Experimental Results

In order to verify the effectiveness of the proposed fingerprint recognition algorithm combining global and local features, the following experiments were carried out.

**Experiment 1 .**

Intra- and interclass sample distance distribution density curve. Thresholds of *R*_1_ and *R*_2_ were determined according to the intra- and interclass sample distance distribution density curves. The collected sample database image was trained, and the Euclidean distances of all intra- and interclass images were calculated. The samples with the corresponding distances form the intra- and interclass sample distance distribution density curve, as shown in Figure 11. The interclass sample indexing density corresponding to *R* < 2.076 is 0. Similarly, the intraclass sample distribution density corresponding to *R* > 3.493 is 0. Therefore, the values of *R*_1_ and *R*_2_ are 2.076 and 3.493, respectively.

RETRACTED

**Experiment 2 .**

Comparison of different methods. The proposed serial matching fusion method was compared with PCA global feature recognition, LBP operator, and traditional fusion based on fractional fusion. The recognition time and recognition rates are shown in Table 3. The proposed global + local serial fusion strategy achieved the highest recognition rate, and it was also superior to local feature recognition and fractional weighted fusion in average recognition speed.

## 6. Conclusions

Global and local features of finger knuckle print represent different features of the image. Global features describe the overall feature and are more suitable for rough extraction. Local features describe image details and are suitable for detail recognition. Therefore, combining the advantages of global features and local features in image recognition helps the recognition of finger knuckle print. Global features with low dimensions were extracted through PCA, which had high recognition speed. According to the experiment results, the four-finger finger knuckle print has different classification weights and contribution rates for the recognition results. The equal-weight distribution method of the existing research was improved. Local features were extracted through the IBP operator. The serial matching fusion strategy was adopted in the fusion of global and local features. The first-layer classifier mainly completed the global feature matching. The samples were initially screened according to the matching result, and all the images in the database were sorted based on the similarity degree. The number of samples to be matched was reduced, and the samples with larger differences were excluded. The second-layer classifier further identified the remaining samples to be matched according to the extracted local features and determined the recognition result. In this paper, a new method based on weighted PCA and LBP is proposed for the first time, and a data set of knuckle and ROI images is established. The proposed algorithm is verified by the data set. In this way, the number of times of fine matching was decreased, and the recognition speed was improved substantially.

RETRACTED

## Figures and Tables

**Figure 1:** Schematic diagram of finger knuckle print and ROI image: (a) finger knuckle print image and (b) ROI image of near finger knuckle print image.

**Figure 2:** Some examples of image in the database: (a) index finger, (b) little finger, (c) middle finger, and (d) ring finger.

**Figure 3:** Relation of cumulative contribution rate and the feature dimension.

**Figure 4:** The knuckle image reconstructed from feature vectors.

**Figure 5:** Schematic diagram of the feature image generation.

**Figure 6:** Relationship between recognition rate and feature dimension: (a) weight ratio 1:1:1:1 and (b) weight ratio 2:3:3:2.

**Figure 7:** Illustration of LBP (8, 2) operator.

**Figure 8:** The ROI images of finger knuckle prints under different light conditions: (a) histogram characteristics of the same samples under light conditions and (b) histogram characteristics of two different collected samples.

**Figure 9:** Comparison of LBP histogram: (a) histogram characteristics of the same samples under light conditions and (b) histogram characteristics of two different collected samples.

**Figure 10:** Schematic diagram of the serial matching strategy of global and local fusion.

**Figure 11:** Intra- and interclass sample distance distribution density curves.

**Table 1:** Experimental results of different weight combinations.

Index	Little	Middle	Ring	Feature dimension
1	1	1	1	32
1	1	2	1	24
1	1	3	2	27
1	2	2	1	22
1	2	3	1	28
1	2	3	2	26
1	3	3	1	24
1	3	3	2	25
1	3	3	2	30
2	1	2	1	26
2	1	3	2	28
2	2	2	1	26
2	2	3	1	24
2	2	3	2	21
2	3	2	1	25
2	3	3	1	24
2	3	3	2	24
3	2	3	1	24
3	2	3	2	25
3	3	2	2	24

**Table 2:** Recognition rate and run time of different LBP operators.

(*P*, *R*)	Recognition rate (%)	Training time (S)	Test time (S)
(8, 1)	90.9	25.40	40.47
(8, 2)	92.4	24.80	40.68
(8, 3)	91.4	25.20	41.02
(16, 1)	88.1	35.21	64.54
(16, 2)	91.6	36.43	66.83
(16, 3)	90.7	36.28	66.54

**Table 3:** Comparison of different methods.

Different methods	Average recognition time of a single image (S)	Recognition rate (%)
PCA	0.028	94.4
LBP	0.149	92.4
Traditional fusion based on score weighting	0.244	98.9
Global + local serial fusion strategy	0.079	99.6

## Data Availability

The image data that support the findings of this study are available from the corresponding author upon reasonable request.
